RETRACTED

# F-box and WD repeat domain-containing 7 (FBXW7) mediates the hypoxia inducible factor-1α (HIF-1α)/vascular endothelial growth factor (VEGF) signaling pathway to affect hypoxic-ischemic brain damage in neonatal rats

**DOI:** 10.1080/21655979.2021.2011635

**Published:** 2021-12-24

**Authors:** Ling Sun

**Affiliations:** Neonatal Intensive Care Unit, Yantaishan Hospital, Yantai, China

**Keywords:** FBXW7, HIF-1α, VEGF, HIBD, angiogenesis

## Abstract

The aim of this study was to determine whether F-box and WD repeat domain-containing 7 (FBXW7) can mediate the hypoxia inducible factor-1α (HIF-1α)/vascular endothelial growth factor (VEGF) signaling pathway to affect neonatal hypoxic-ischemic brain damage (HIBD) in neonatal rats. HIBD rats were treated with LV-shFBXW7. Cerebral infarct size was determined by 2,3,5-triphenyltetrazolium chloride (TTC) staining, while microvessel density (MVD) was evaluated by immunohistochemistry. Learning and memory were tested using the Morris water maze (MWM) test. FBXW7 and HIF-1α/VEGF signaling pathway proteins were measured by Western blotting. Brain microvascular endothelial cells (BMECs) were isolated to establish an oxygen-glucose deprivation (OGD) model to evaluate treatment with FBXW7 siRNA. Cell viability was detected using a 3-[4,5-dimethylthiazol-2-yl]-2,5 diphenyl tetrazolium bromide (MTT) assay, while cell migration was evaluated using a wound healing assay. The tube formation of BMECs was also assessed. The results demonstrated that HIBD rats exhibited increased protein expression of FBXW7, HIF-1α, and VEGF. HIBD rats also displayed increased cerebral infarct size, prolonged escape latency and a decreased number of platform crossings. However, HIBD rats treated with LV-shFBXW7 exhibited reversal of these changes. *In vitro* experiments showed that BMECs in the OGD group had significantly decreased cell viability, shorter vascular lumen length, and shorter migration distance than cells in the control group. Moreover, silencing FBXW7 promoted proliferation, tube formation and migration of BMECs. Taken together, silencing FBXW7 upregulates the HIF-1α/VEGF signaling pathway to promote the angiogenesis of neonatal HIBD rats after brain injury, reducing infarct volume and improving recovery of nerve function in HIBD rats.

## Introduction

Neonatal hypoxic-ischemic brain damage (HIBD) is brain injury after perinatal asphyxia and hypoxia during the neonatal period [1], which not only poses a serious threat to the health of neonates but has also become a major cause of neonatal death and childhood disability [2]. To date, the pathophysiological mechanism of HIBD remains to be investigated. Many factors in recent studies have been reported to contribute to HIBD, such as excitatory amino acid-induced toxicity, calcium overload and inflammation [1,3]. At present, many treatments and intervention methods for neonatal HIBD tend to have limitations or side effects and cannot radically prevent the occurrence of neurological sequelae, which means that the clinical effect of these therapies is far from satisfactory [4,5]. Thus, further understanding of the precise mechanisms involved in neonatal HIBD and identifying new targets for the prevention and treatment of HIBD are of great significance for improving quality of life in neonates.

RETRACTED

Encoded by the F-box and WD repeat domain-containing 7 (FBXW7) gene, the FBXW7 protein is a member of the F-box protein family and is widely distributed in human tissues and cells [6]. Several studies have presented evidence that FBXW7 acts as a widespread tumor suppressor in cellular processes, such as proliferation, growth, and apoptosis [7,8]. In addition, FBXW7 has also been shown to play vital roles in vascular endothelial cell migration and inflammation, as well as endothelial barrier integrity, angiogenesis and the formation of atherosclerotic plaques [9,10]. For instance, Chen *et al*. reported that miR-322 reduces cardiomyocyte apoptosis and infarct size by targeting FBXW7, contributing to protecting the heart from myocardial ischemia/reperfusion-induced injury [11]. Additionally, FBXW7 was revealed to regulate neuronal apoptosis during the progression of spinal cord injury (SCI) by mediating microglial inflammation in a study of Chen *et al*. [12]. However, it has not been reported whether FBXW7 is involved in neonatal HIBD. Coincidentally, Cassavaugh *et al*. found that FBXW7 regulates angiogenesis in hypoxic cells through the targeted regulation of hypoxia inducible factor-1α (HIF-1α) expression [13]. In addition, vascular endothelial growth factor (VEGF) is one of the most important target genes of HIF-1α during hypoxia [14]. In response to ischemia and hypoxia, HIF-1α activates transcription of the VEGF gene to increase VEGF levels and promote angiogenesis, improving blood supply to ischemic tissues [15].

FBXW7 recognizes phosphorylated HIF-1α and mediates its ubiquitination and degeneration [16]. Of note, Ga Won Jeon *et al*. reported that HIF-1α deficiency aggravates neonatal hypoxic-ischemic injury [17]. Given these findings, we hypothesized that FBXW7 regulates the HIF-1α/VEGF pathway to affect neonatal HIBD. Herein, this study attempted to elucidate the involvement of FBXW7 in neonatal HIBD models through the HIF-1α/VEGF pathway, hoping to provide a new perspective for the treatment of neonatal HIBD.

## Materials and methods

### Ethics statement

This study was conducted in accordance with the *Guide for the Care and Use of Laboratory Animals* [18] and was approved by the Medical Ethics Committee of Laboratory Animals in our hospital.

RETRACTED

### Preparation of the HIBD rat model

The HIBD rat model was successfully established as previously described [19]. In brief, rats were anesthetized with 3% isoflurane and fixed on a thermostatic operation table in the supine position. The neck area for surgery was routinely disinfected with iodophor and alcohol. Ophthalmic scissors were used to cut the skin slightly to the right along the median line of the rat’s neck, exposing and separating the right common carotid artery (RccA) without damaging the right vagus nerve. The proximal and distal ends of the RccA were ligated, and the middle of the two ligation points was sliced. The incision was sutured and disinfected. After surgery, pups were allowed to recover for 1 h at 37°C and were then exposed to hypoxia (92% N_2_ + 8% O_2_) at 36 ± 6°C for 2.5 h. Pups were returned to lactating dams. Sham-operated rats were only subjected to isolation and ligation of the common carotid artery without occlusion or hypoxia. Six, 12, 24, and 48 h after model establishment, FBXW7 expression in the brain tissues of 6 rats from each group was assessed.

### Experimental animal grouping

Rats were divided into four groups: sham, HIBD, HIBD + LV-shNC and HIBD + LV-shFBXW7, with 12 rats in each group. Forty-eight hours before model establishment, rats in the HIBO + LV-shNC and HIBO + LV-shFBXW7 groups were intracerebroventricularly (ICV) injected with LV-shNC/LV-shFBXW7 (coordinates: 2 mm posterior, 2 mm lateral, and 3 mm below the skull surface) [20]. Lentiviral vectors expressing FBXW7 shRNA (LV-sh-FBXW7, 5ʹ-TAAAGAGTTGGCACTCTAT-3ʹ) and negative control shRNA (LV-shNC, 5ʹ-TTCTCCGAACGTGTCACGT-3ʹ) were designed and synthesized by Shanghai GenePharma Co., Ltd. The detailed experimental protocol is illustrated in Figure 1.

**Figure 1.** *In vivo* experimental diagram

### Triphenyl tetrazolium chloride (TTC) staining

Forty-eight hours after model establishment, the infarct size of rats was determined using TTC staining [21]. In brief, six rats in each group were anesthetized and rapidly decapitated to obtain the brain, with the olfactory bulb, cerebellum and lower brainstem removed. The brain was frozen at −20°C for 15–20 min. Serial brain sections of 2-mm thickness were stained in 2% TTC at 37°C for 20 min, washed with PBS, and then immersed overnight in 4% paraformaldehyde. The next day, the stained slices were collected for imaging, and the infarct volume was analyzed using ImageJ software.

### Hematoxylin and eosin (HE) staining

Pathological damage to brain tissues was assessed using HE staining [22]. Briefly, rat brain sections were fixed in 4% paraformaldehyde for at least 24 h, dehydrated and embedded in paraffin. After slicing, serial 5-μm brain sections were immersed in xylene I and II for 10 min for deparaffinization, followed by 100% ethanol for 2 min, 95% ethanol for 1 min, 80% ethanol for 1 min, 75% ethanol for 1 min and distilled water for 2 min. Next, brain sections were stained with hematoxylin for 5–7 min, washed with tap water, reblued with 1% hydrochloric alcohol, washed with tap water, and counterstained with eosin for 3 min prior to routine procedures, such as dehydration, hyalinization and sealing with neutral resin.

RETRACTED

### Examination of cerebral cortical microvessel density (MVD) in rats

MVD was evaluated by immunohistochemistry [23]. Brain tissues of rats were fixed in 10% formaldehyde, embedded in paraffin, sliced into tissue sections, deparaffinized and rehydrated. Tissue sections were immersed in antigen retrieval solution, placed in an autoclave for 15 min, allowed to cool naturally at room temperature, and washed with PBS 3 times for 3 min each. Next, 3% H_2_O_2_ was dropped onto tissue sections, which were kept in the dark for 10 min to block the activation of endogenous peroxidase. Then, the anti-CD31 primary antibody (Abcam, UK) was added overnight at 4°C, followed by horseradish peroxidase (HRP)-labeled secondary antibodies at room temperature for 30 min. Diaminobenzidine (DAB) chromogenic solution was added dropwise, and neutral resin was used for sealing. Tissue sections were observed and imaged under a microscope, and MVD in the cerebral cortex was quantified.

### Terminal-deoxynucleotidyl transferase nick end labeling (TUNEL) staining

Neuronal apoptosis in the hippocampal CA1 region was examined using the TUNEL assay (Roche, CA, USA) according to the manufacturer’s instructions [24]. Coronal sections were obtained from the middle region of the optic chiasm and papillary body. Apoptotic neurons in the hippocampal CA1 area were observed in five random visual fields by microscopy. Apoptotic cells were counted using Image-Pro Plus image analytic software (Media Cybernetics, USA).

### Assessment of inflammatory markers

The concentrations of various proinflammatory cytokines, such as interleukin-1β (IL-1β), interleukin-6 (IL-6), and tumor necrosis factor-alpha (TNF-α), in cerebral homogenates were assessed using commercially available enzyme-linked immunosorbent assay (ELISA) kits following the protocols provided by the manufacturer (Thermo Fisher Scientific Inc., MA, USA) [25].

### Morris water maze (MWM) test

Each group had 6 rats that were fed until 4 weeks old for the MWM test, which was performed as previously described [26]. Platform navigation testing lasted 5 days. On each day, rats were placed in the water face-down from randomly selected sites in the four quadrants, and the escape latency, namely, the time spent finding and climbing on the platform, was recorded. If the rat did not locate the platform within 120 s, it was placed on the platform and allowed to stay there for 10 s. In this case, the escape latency was recorded as 120 s. Rats were trained 4 times a day, and the mean escape latency was used to evaluate leaning ability. A spatial probe test was conducted 24 h after the platform navigation test. The platform was removed, and the rat was placed into the water from a randomly selected entry site. The number of platform crossovers within 120 s was recorded, and the mean value of 4 tests each day was used to evaluate the memory of rats.

RETRACTED

### Quantitative reverse transcriptase polymerase chain reaction (qRT–PCR)

The silencing efficiency of FBXW7 was confirmed using qRT–PCR [27]. Total RNA was isolated using TRIzol reagent (Thermo Fisher, USA). Next, 1 μg of total RNA was used to synthesize cDNA with the cDNA Synthesis Kit (Thermo Fisher, USA). Finally, PCR was performed using a QuantiTect Multiplex RT–PCR Kit (QIAGEN, Germany) to analyze the expression of FBXW7. Primers used for qRT–PCR were synthesized by Shanghai Biological Engineering Technology Services Co. Ltd. (Shanghai, China): FBXW7 forward: 5ʹ-GTTCCGCTGCCTAATCTTCCT-3ʹ and reverse: 5ʹ-CCCTTCAGGGATTCTGTGCC-3ʹ; GAPDH forward: 5ʹ-AATGGATTTGGACGCATTGGT-3ʹ and reverse: 5ʹ-TTTGCACTGGTACGTGTTGAT-3ʹ. Relative expression was determined using GAPDH as an internal control and reported as 2^−ΔΔCT^.

### Western blotting

Western blotting analysis was performed as previously reported [28]. Whole-cell lysates were used to extract proteins from rat brain tissues in radioimmunoprecipitation assay (RIPA) lysis buffer and were quantified for protein concentration using a bicinchoninic acid (BCA) kit. The protein sample was mixed with the loading buffer and heated in a boiling water bath for denaturation. The same concentration of denatured protein sample was added to each loading well. Proteins were separated using 10% sodium dodecyl sulfate–polyacrylamide gel electrophoresis (SDS–PAGE) and transferred onto polyvinylidene fluoride (PVDF) membranes using a semidry transfer system (Bio–Rad, USA). After blocking in defatted milk powder for 1 h at room temperature, the membranes were washed with phosphate buffer solution with Tween 20 (PBST) and incubated overnight at 4°C with primary antibodies against FBXW7, HIF-1α VEGF and GAPDH (all purchased from Abcam). Next, the membranes were washed with PBST (5 times × 3 min) and incubated with HRP-secondary antibodies for 1 h. Blots of target proteins were developed using an enhanced chemiluminescence (ECL) kit. Using GAPDH as the loading control, the relative expression of target proteins is expressed as the gray value ratio of the target protein to GAPDH.

RETRACTED

### Culture of brain microvascular endothelial cells (BMECs)

BMEC isolation was performed as previously described [29]. Postnatal SD rats were anesthetized and decapitated to obtain the cerebral cortex, which was cut into 1 cm^3^ pieces using ophthalmic scissors. The cerebral cortex was minced, and the homogenate was filtered through 80-mesh and 200-mesh filter screens. The filtrate (microvascular segment) was collected and digested in 10 mL 0.2% collagenase II at 37°C for 20 min, followed by centrifugation at 1000 r/min for 5 min. The precipitate was washed with endothelial cell flushing solution 3 times and centrifuged. Cells were resuspended and seeded into culture flasks precoated with gelatin for incubation at 37°C and 5% CO_2._ The culture medium was renewed 48 h after cells were plated and every 3 days thereafter. When cell confluence reached 75%–85%, cells were passaged to the third generation and collected for subsequent experiments.

### Establishment and grouping of oxygen-glucose deprivation (OGD) model rats

BMECs were divided into four groups: control, OGD, OGD + siNC, OGD + siFBXW7-1, and OGD + siFBXW7-2. Cells in the OGD group were placed in an anaerobic chamber (BINGDER150, Germany) with 5% CO_2_ and 95% N_2_. Normal culture medium was replaced with deoxygenated, glucose-free Earle’s balanced salt solution (EBSS) to expose cells to the OGD environment at 37°C for 4 h [30]. Cells in the control group were cultured in a conventional CO_2_ incubator. Cells in the OGD + siNC, OGD + siFBXW7-1 and OGD + siFBXW7-2 groups were transfected with NC siRNA (5ʹ‑UUCUCCGAACGUGUCACGUUU‑3ʹ) and FBXW7-1 siRNA (5ʹ‑ACAGGACAGUGUUUACAAA‑3ʹ) and FBXW7-2 siRNA (5ʹ‑CCAUGCAAAGUCUCAGAAU‑3ʹ) (all purchased from Shanghai GenePharma Co., Ltd), respectively, before exposure to the OGD environment. Cell transfection was conducted according to the instructions of the Lipofectamine 2000 kit (Invitrogen, USA). After trypsin digestion, BMECs were collected in logarithmic growth phase, resuspended, counted and seeded into 12-well plates (5 × 10^4^ cells/well). Plates were gently oscillated to evenly distribute the cells. Cells were cultured at 37°C and 5% CO_2,_ and transfection was performed the next day when cell confluence had reached 70%–80%.

### 3-[4,5-Dimethylthiazol-2-yl]-2,5 diphenyl tetrazolium bromide (MTT) assay

The MTT assay was conducted according to a previously described method [31]. Cells in each group were inoculated into 96-well plates at 1 × 10^4^ cells/well and cultured at 37°C and 5% CO_2_. After the required intervention, 10 μL MTT (5 mg/mL) was added to each well and incubated at 37°C for 4 h. Then, the upper supernatant was discarded, and 100 μL dimethylsulfoxide (DMSO) was added to each well for 10 min of gentle oscillation until the full dissolution of purple black crystals. The optical density (OD) value of each well was measured at 450 nm using a microplate reader. Cell viability (%) = (OD value _Model group_ – OD value _Blank group_)/(OD value _Control group_ – OD value _Blank group_) × 100%. The experiment was conducted three times.

RETRACTED

### Tube formation assay

The tube formation assay was performed based on a previous study [32]. Before the experiment, BD Matrigel without growth factor was kept at 4°C overnight for dissolution, and 200 μL pipette tips and 96-well plates were precooled overnight at −20°C. The next day, 100 μL of precooled Matrigel was added to 96-well plates (to prevent bubbles) and incubated for 30 min at 37°C. After trypsin digestion, BMECs were collected in logarithmic phase and seeded into 96-well plates (1 × 10^4^ cells/well). Plates were gently oscillated for even distribution of cells, which were cultured at 37°C and 5% CO_2._ After 16 h, tube formation was assessed using an inverted microscope.

### Wound healing assay

The wound healing assay was performed following a published method [33]. BMECs were seeded into Ibidi dishes with a culture insert (Ibidi, Germany) at 3 × 10^5^ cells/well and cultured at 37°C and 5% CO_2._ After overnight incubation, the inserts were removed using sterile forceps, and a 500 µm-wide line was created in the cell monolayer. The plate was washed with PBS to remove detached cells and observed and imaged under an inverted Leica microscope (0 h). Cells were cultured for 12 h and observed, with 5 different visual fields imaged under an inverted Leica microscope (12 h). WimScratch software (Ibidi, Germany) was used to analyze the migration distance of cells.

### Statistical methods

All statistical data were analyzed using SPSS 21.0 software (SPSS, Inc., Chicago, IL, USA). Measurement data are shown as the mean ± standard deviation (SD). Differences among multiple groups were compared using one-way ANOVA, while comparisons between two groups were analyzed using post hoc Tukey’s test. Differences were considered significant if *P* < 0.05.

## Results

### Expression of FBXW7 and the HIF-1α/VEGF signaling pathway in brain tissues of HIBD rats

To explore the function of FBXW7 and HIF-1α/VEGF in HIBD, we established an HIBD model in rats. Western blotting was conducted to determine the expression of FBXW7 and HIF-1α/VEGF signaling pathway proteins in HIBD rats. Consequently, FBXW7 expression was significantly higher in the brain tissues of HIBD model rats than in sham group rats and peaked 48 h after HIBD (all *P* < 0. 05). Similarly, protein levels of HIF-1α and VEGF were increased in the HIBD group compared to the sham group (both *P* < 0. 05), peaking at 24 h and beginning to decline at 48 h (Figure 2). Thus, these data suggested that FBXW7 and HIF-1α/VEGF are involved in brain injury in HIBD rats.

RETRACTED

**Figure 2.** Expression of the F-box and WD repeat domain-containing 7 (FBXW7) and hypoxia inducible factor-1α (HIF-1α)/vascular endothelial growth factor (VEGF) signaling pathways in brain tissues of hypoxic-ischemic brain damage (HIBD) rats

Note: a, Western blotting analysis of FBXW7 and the HIF-1α/VEGF signaling pathway in HIBD rats 6, 12, 24, and 48 h after model establishment. b-d, Expression of FBXW7 (b), HIF-1α (c) and VEGF (d) in HIBD rats 6, 12, 24, and 48 h after model establishment. The data are shown as the mean ± standard deviation (SD) (n = 6). *P < 0.05, versus sham group.

### Effect of FBXW7 silencing on infarct size, angiogenesis, and apoptosis in HIBD brains

Cerebral infarct size in the brain was assessed using TTC staining. The results revealed that the HIBD group had a significantly larger cerebral infarct size than the sham group, while the cerebral infarct size of the HIBD + LV-shFBXW7 group was notably decreased compared with that of the HIBD group all *P* < 0. 05, Figure 3(a-b). Histopathological changes in the HIBD brain tissues were assessed by HE staining. The results showed that in the HIBD group, cerebral cortex structure was disordered, and histological stratification disappeared with the loose empty network Figure 3(c), but cerebral damage was effectively alleviated in rats in the HIBD + LV-shFBXW7 group. Immunohistochemical staining of CD31 was next used to evaluate MVD Figure 3(d). HIBD rats exhibited increased cerebral cortical MVD compared to sham rats, while the HIBD + LV-shFBXW7 group displayed significantly increased cerebral cortical MVD compared to the HIBD group all *P* < 0. 05, Figure 3(f). TUNEL staining results Figure 2(e) revealed that the sham group presented a small amount of apoptosis in the hippocampal CA1 region. Compared to the sham group, the HIBD group exhibited an increased apoptosis rate (*P* < 0.05). In contrast, the HIBD + LV-shFBXW7 group displayed a decreased apoptosis rate compared to the HIBD group (*P* < 0.05). These findings supported that silencing FBXW7 alleviates brain injury and promote angiogenesis in HIBD rats.

RETRACTED

**Figure 3.** Effect of FBXW7 silencing on infarct size, angiogenesis, and apoptosis in HIBD brains

Note: a-b: Cerebral infarct size of neonatal rats in each group was evaluated using 2,3,5-triphenyltetrazolium chloride (TTC) staining. c, Pathological changes in the cerebral cortex in neonatal rats were observed by hematoxylin-eosin (HE) staining; black arrows indicate infiltrated inflammatory cells. d, Cerebral cortical microvessel density (MVD) was evaluated by immunohistochemical staining; black arrows indicate CD31-positive vessels. e, Terminal-deoxynucleotidyl transferase nick end labeling (TUNEL) staining of rat hippocampal sections with arrows indicating TUNEL-positive cells. f, Quantitative determination of mean CD31-positive vessel numbers of rats in each group. g, Apoptosis rate of the hippocampal CA1 region of rats in each group. All data shown are the mean ± SD (n = 6). *P < 0.05, versus sham group; #*P* < 0.05, versus HIBD group.

### Effect of FBXW7 silencing on neuroinflammation, learning and memory in HIBD rats

The levels of inflammatory cytokines were measured using ELISA Figure 4(a). The results revealed upregulated levels of the inflammatory cytokines IL-1β, TNF-α and IL-6 in the HIBD group (all *P* < 0. 05). Treatment with shFBXW7 significantly decreased HIBD-induced increases in these inflammatory cytokines (all *P* < 0. 05). The MWM test was used to assess learning and memory in rats. Rats in the HIBD group demonstrated significantly longer escape latency and remarkably fewer platform crossings than those in the sham group (both *P* < 0. 05). Compared to the HIBD group, rats in the HIBD + LV-shFBXW7 group exhibited a prominently decreased escape latency and a remarkable increase in the number of platform crossings both *P* < 0. 05, Figure 4(b-d). Given the above findings, silencing FBXW7 significantly attenuates neuroinflammation and improves learning and memory in HIBD rats.

**Figure 4.** Effect of FBXW7 silencing on neuroinflammation, learning and memory in HIBD rats

Note: a, Levels of inflammatory cytokines, including tumor necrosis factor-alpha (TNF-α), interleukin-1β (IL-1β) and interleukin-6 (IL-6), were detected using enzyme-linked immunosorbent assay (ELISA) on rats in each group. b, Platform navigation test in the Morris water maze test (MWM) was used to examine escape latency of rats. c, Spatial probe trial of MWM was used to measure the number of platform crossings. d, Swimming traces of neonatal rats in each group. Results are expressed as the mean ± SD (n = 6). *P < 0.05, versus sham group; #*P* < 0.05, versus HIBD group.

RETRACTED

### Expression of FBXW7 and HIF-1α/VEGF pathway proteins in brain tissues of HIBD rats

According to the qRT–PCR results, rats in the HIBD + LV-shFBXW7 group exhibited 70.19% FBXW7 mRNA silencing efficiency compared to the HIBD group Figure 5(a). Protein expression of FBXW7 and the HIF-1α/VEGF pathway in the brain tissues of rats was assessed by Western blotting Figure 5(b-e). HIBD rats had prominently increased protein expression of FBXW7, HIF-1α and VEGF compared to sham group rats (all *P* < 0. 05). Meanwhile, rats in the HIBD + LV-shFBXW7 group had significantly reduced FBXW7 expression and notably elevated HIF-1α and VEGF protein expression compared to HIBD rats (all *P* < 0. 05). Thus, silencing FBXW7 activates the HIF-1α/VEGF signaling pathway.

**Figure 5.** FBXW7 and the HIF-1α/VEGF pathway protein expression in brain tissues of HIBD rats

Note: a, FBXW7 mRNA in rat brain tissues was detected by quantitative reverse transcriptase polymerase chain reaction (qRT–PCR). b, Protein expressions of FBXW7 and HIF-1α/VEGF pathway in brain tissues of rats was assessed by Western blotting. c-e, Comparison of protein expression of FBXW7, HIF-1α and VEGF in brain tissues from rats in different groups. The data are shown as the mean ± SD (n = 6). * *P* < 0.05, versus sham group; # *P* < 0.05, versus HIBD group.

### FBXW7 regulates the function and angiogenesis of BMECs in vitro

MTT, tube formation, and wound healing assays were conducted to determine proliferation, tube formation and migration, respectively, in BMECs (Figure 6). BMECs in the OGD group displayed markedly reduced cell viability, fewer vascular lumen-like structures, and shorter tube length and migration distances than cells in the control group (all *P* < 0. 05). Compared to the OGD group, BMECs from the OGD + siFBXW7 group exhibited increased cell viability, more vascular lumen-like structures, longer tube length and greater migration distance (all *P* < 0. 05). These findings supported that silencing FBXW7 promotes proliferation, tube formation and migration in BMECs.

**Figure 6.** FBXW7 regulates the function and angiogenesis of brain microvascular endothelial cells (BMECs) *in vitro.*

Note: a, Cell viability of BMECs as determined by 3-[4,5-dimethylthiazol-2-yl]-2,5 diphenyl tetrazolium bromide (MTT) assay. b, Tube length of BMECs in different groups. c, Migration distance of BMECs in different groups. d, Tube formation ability of BMECs examined by tube formation assay. e, Migration ability of BMECs evaluated by wound healing assay. Error bars represent the mean ± SD of three independent experiments (n = 3). *P < 0.05, versus control group; #*P* < 0.05 versus OGD group.

## Discussion

In this study, we observed significant upregulation of FBXW7, HIF-1α and VEGF in the brain tissues of rats after HIBD model establishment. In agreement, Weinian Gao *et al*. reported prominently upregulated mRNA and protein expression of FBXW7 in cardiac hypertrophy in mice and angiotensin II (ANG II)-induced hypertrophic neonatal rat cardiomyocytes (NRCMs) [27]. Another study by Wenzhi Tan *et al*. identified increased FBXW7 expression in intestinal ischemia-reperfusion (I/R) injury; however, FBXW7 deletion alleviated apoptosis of intestinal epithelial cells [34]. On the other hand, focal cerebral ischemia model mice, as established by F Shen *et al*., displayed upregulated HIF-1α expression in the ischemic area and elevated VEGF expression in the ischemic perifocal region, with increased total numbers of microvessels and newly formed microvessels, which promote the recovery of injured nerves after ischemia [35]. As evidenced by a previous study, ischemia and hypoxia cause degeneration, necrosis and apoptosis of nerve cells, resulting in damage to nerve functions [36]. Hence, it is of critical importance for the recovery of neurological function to restore blood supply to the ischemic area as soon as possible [37,38]. Angiogenesis is a complex process involving the generation of new capillaries from preexisting blood vessels and is an effective way to improve blood supply to brain tissues [39]. VEGF was suggested to be the strongest factor promoting angiogenesis and can bind to the VEGF receptor to stimulate the differentiation and maturation of precursors of vascular endothelial cells, promoting the migration and adhesion of vascular endothelial cells [40,41]. The promoter region of the VEGF gene has a binding site for HIF-1α, and its combination with HIF-1α under ischemic and hypoxic conditions induces gene expression of VEGF [42,43]. Therefore, the upregulated expression of HIF-1α and VEGF after neonatal HIBD may result from adaptive and protective changes in cells and tissues in a hypoxic environment, which is conducive to angiogenesis and neural repair. Of note, Daniela Flügel *et al*. revealed that FBXW7 and USP28 reciprocally regulate the migration and angiogenesis of cells in a HIF-1α-dependent manner [44]. Given these findings, FBXW7 may play a regulatory role in neonatal HIBD by mediating the HIF-1α/VEGF pathway.

RETRACTED

Next, FBXW7 was inhibited in HIBD rats in our subsequent experiments, and as a consequence, the cerebral infarction area was reduced with promoted angiogenesis and improved learning and memory in HIBD rats. In a similar vein, Mi Yang *et al*. demonstrated that miR-497-195 maintains HIF-1α stability to increase angiogenesis and reduce bone loss by targeting FBXW7 [45], indicating that FBXW7 protects the brain of neonatal HIBD rats by promoting angiogenesis and reducing the cerebral infarction area. The primary mechanisms of neonatal HIBD include oxidative stress, excitability, inflammation, and apoptosis [46]. There is considerable evidence indicating that apoptosis plays an important role in the evolution and propagation of HIBD [21]. Furthermore, proinflammatory cytokines (IL-6, TNF-α, and IL-1β) induce microglial activation, which favors the production of additional cytokines and a subsequent inflammatory cascade [47]. In the present study, pretreatment of rats with shFBXW7 significantly inhibited HIBD-induced apoptosis, reduced levels of proinflammatory cytokines, and further repaired neuronal injury. Accordingly, we concluded that FBXW7 silencing exerts neuroprotective effects in HIBD.

Another important finding of the current study was that silencing FBXW7 further upregulates HIF-1α and VEGF expression levels in the brain tissues of HIBD rats. Coincidentally, Cassavaugh *et al*. also reported that silencing FBXW7 in hypoxia reduces ubiquitinated HIF-1α levels to improve HIF-1α expression [13]. Additionally, Cur20 enhanced angiogenesis in model mice with cerebral ischemic injury by activating the HIF-1α/VEGF signaling pathway, notably attenuating cognitive dysfunction in mice [48]. As revealed by Rania G Abdel-Latif *et al*., empagliflozin upregulates the expression of the HIF-1α/VEGF signaling pathway to reduce the cerebral infarction area and alleviate neuronal apoptosis and cerebral injury in I/R-injured rats [49]. Many studies have shown that upregulation of HIF-1α can be induced by overexpression of VEGF in ischemic brain injury, which can, on the one hand, alleviate brain injury after ischemia by promoting the proliferation and migration of microvascular endothelial cells (MECs), increasing angiogenesis, improving local blood supply, and protecting endothelial cells from degeneration and necrosis, while at the same time protecting neurons by directly or indirectly inhibiting neuronal apoptosis [50–52]. All of these findings support that silencing FBXW7 upregulates the HIF-1α/VEGF pathway to promote angiogenesis and protect neurons in neonatal HIBD rats.

As previously reported, the proliferation and migration of vascular endothelial cells and the formation of capillary-like structures are important steps in angiogenesis [53]. In the present study, BMECs were isolated, and an *in vitro* OGD model was established to mimic cerebral ischemic/hypoxic injury. Proliferation, tube formation and migration abilities in BMECs were remarkably improved after silencing FBXW7. Similarly, Hongjin Wang *et al*. also observed that catalpol promotes proliferation, migration and tube formation in BMECs by activating the HIF-1α/VEGF pathway, ultimately attenuating OGD-induced injury of BMECs [30]. Daniela Flügel *et al*. reported that silencing FBXW7 increased cell migration and angiogenesis via the mediation of HIF-1α expression [44]. All of these findings further demonstrate that silencing FBXW7 promotes angiogenesis by enhancing the proliferation and migration of vascular endothelial cells, alleviating hypoxia/ischemia-induced brain injury. However, there was a limitation in this study. Due to time limitations and experimental conditions, we did not use two shRNAs in the animal study to confirm the target-specific effect of silencing. Thus, more complete studies are still needed in the future.

RETRACTED

## Conclusions

In summary, our data showed that silencing FBXW7 upregulates the HIF-1α/VEGF signaling pathway to promote angiogenesis after brain injury, reducing the cerebral infarction area and promoting neurological function recovery in neonatal HIBD rats. In this regard, this study may offer a new theoretical basis for the treatment of neonatal HIBD.
